# Characterization of the anti-*Staphylococcus aureus* fraction from *Penthorum chinense* Pursh stems

**DOI:** 10.1186/s12906-019-2632-3

**Published:** 2019-08-17

**Authors:** Bin Ding, Qinchao Ding, Shun Zhang, Zhuo Jin, Zhaolei Wang, Songtao Li, Xiaobing Dou

**Affiliations:** 1 Zhejiang Chinese Medical University, No. 548 Binwen Road, Hangzhou, 310053 Zhejiang People’s Republic of China; 2 Ningbo No.2 Hospital, Ningbo, 315010 People’s Republic of China

**Keywords:** *Staphylococcus aureus* (*S. aureus*), *Penthorum chinense* pursh, Bacteriostatic activity, Bactericidal activity

## Abstract

**Background:**

Methicillin-resistant *Staphylococcus aureus* (MRSA) causes serious infections in hospitals. *Penthorum chinense* Pursh (PCP), employed by the Miao ethnic minority in China, presents antibacterial activities. In this study, the anti-*Staphylococcus aureus* activities in the pinocembrin-7-O residue-rich fraction from PCP (PGF) were evaluated and characterized.

**Methods:**

The PGF was prepared with 70% ethanol reflux extraction followed by fractional extraction and column chromatography. Pinocembrin-7-O residue components were identified with electrospray ionization mass spectrometry (ESI-MS). Anti-*S. aureus* activities of the fraction and the main components were evaluated in vitro with serially diluted microbroth assays. Cytotoxicity was evaluated with 3-(4,5-dimethylthiazol-2-yl)-2,5-diphenyltetrazolium bromide (MTT) chromogenic assays using the NCTC 1469 cell line.

**Results:**

This study indicated that the PGF and three components (S1, S2, and S3) presented anti-*S. aureus* activities, including against clinically isolated MRSA strains. The molecular masses of S1, S2, and S3 were identical to those of pinocembrin-7-O-[4″,6″-hexahydroxydiphenoyl (HHDP)]-β-D-glucose, pinocembrin-7-O-[3″-O-galloyl-4″,6″-(s)-HHDP]-β-D-glucose, and Thonningianin A, respectively. The PGF, S1, S2, and S3 all presented an identical minimum inhibitory concentration (MIC) against *S. aureus* ATCC 25923 and ATCC 43300, which was 62.5 μg/mL. The minimum bactericidal concentrations (MBCs) of the PGF and S3 against ATCC 25923 were 125 and 250 μg/mL, and the MBCs of the PGF, S2, and S3 against ATCC 43300 were 250, 500, and 250 μg/mL, respectively. A time-kill assay consistently indicated that none of the bacterial clones of ATCC 25923 and ATCC 43300 could survive under 2× and 4× MIC PGF treatment for 24 h, respectively. In contrast, 10^4^ CFU (colony-forming units) of ATCC 25923 and ATCC 43300 were killed by 8× and 4× MIC S3 within 24 h, respectively. Additionally, 1×, 2×, and 4× MIC the PGF presented similar postantibiotic effects (PAEs) on the strain ATCC 25923. However, the PAE of the PGF on the strain ATCC 43300 was concentration dependent (1× < 2× < 4× MIC). Finally, the PGF (200 μg/mL) and S3 (60 μg/mL) showed no cytotoxicity against human hepatoma cells.

**Conclusions:**

The PGF and S3 from PCP present potential for the treatment of *S. aureus* and MRSA infections. The components S1 and S2 present inhibition activities against *S. aureus*.

## Background

*Staphylococcus aureus*, a gram-positive, facultative anaerobic bacterium with a round shape, is frequently isolated from the skin, eyes, and upper respiratory tract [1]. It is a common opportunistic pathogen and remains a major cause of skin infection. Generally, immunodeficient patients who undergo surgery [2] or have prosthetic implants [3], as well as patients with life-threatening diseases [4], are considered to have a high risk of *S. aureus* infection. *S. aureus* infection may enhance the mortality rate up to 40% [5]. Since antibiotics were discovered, some of them, such as methicillin, have been widely used against *Staphylococcus* infection. However, methicillin-resistant *Staphylococcus aureus* (MRSA) was reported very rapidly. In clinical practice, vancomycin is used normally as an alternative antibiotic for MRSA infection treatment [6]. In recent years, antimicrobial resistance is a significantly increasing problem, and some MRSA strains have developed multidrug resistance capabilities [7–9]. Therefore, novel anti-MRSA agents are urgently needed.

Certain Chinese medical herbs have been employed in the treatment of bacterial or viral infection for a very long time [10]. Gan Huang Cao, *Penthorum chinense* Pursh (Penthoraceae), is used as a functional food and folk medicine by the Miao ethnic minority in China [11]. Miao people prepare meals with young PCP leaflets and drink PCP wine to prevent alcohol hangover symptoms. It was also used in the clinic to treat hepatic viral diseases [12], such as acute hepatitis virus infection, and shows positive effects. A previous study demonstrated that PCP extract could inhibit the growth of *Pseudomonas aeruginosa*, *Staphylococcus aureus*, and *Staphylococcus epidermidis* in vitro [13] and the flavonoids in PCP presented anti-complement activities [14]. Hence, the major flavonoids in PCP have been identified [15, 16]. However, little is known about which component(s) presents the antibacterial capability. In this study, we identified and characterized the anti-*S. aureus* activities of three pinocembrin derivatives in PCP stems.

## Methods

### Bacterial strains

*S. aureus* ATCC 29213, *S. aureus* ATCC 43300, *S. aureus* ATCC 25923, *Lactobacillus rhamnosus* ATCC 53103, and *Streptococcus thermophilus* ATCC 19258 were purchased from the American Type Culture Collection (ATCC, Manassas, VA). *Staphylococcus epidermidis* CMCC26069 and *Bacillus subtilis* CMCC1.1470 were purchased from the China General Microbiological Culture Collection Center (CGMCC, Beijing, China). Seven clinical isolates were identified and characterized by Mr. Shun Zhang (Ningbo No. 2 Hospital, Zhejiang Province, China). The bacteria were grown on Mueller–Hinton (MH) broth on agar plates or in liquid medium.

### Active fraction preparation

Stems of PCP were purchased from Sichuan Chinese Medicine Yinpian Co., Ltd. and identified by Prof. Ding (Zhejiang Chinese Medical University). The dried stems were powdered with an electric herb-grinding machine and sifted with an 80-mesh screen. Powdered stem (250 g) was reflux extracted twice with 2.5 L of 70% ethanol for 1.5 h. This crude extract of PCP was concentrated in a rotary vacuum evaporator. The components in this crude extract were fractionally extracted with petroleum ether, ethyl acetate, 1-butanol and water. All the fractions were vacuum dried, and the concentration of flavonoids was determined with a chromogenic reaction [13]. The 3 g ethyl acetate fraction, dissolved in 30 mL of 30% ethanol, was loaded into a 30% ethanol-equilibrated HPD 500 column (40 × 40 mm) (Guangfu Fine Chemical Research Institute (Tianjin, China)) and washed with 3 column volumes of 30% ethanol. The PGF was eluted with 5 column volumes of 80% ethanol.

### Characterization and identification the components in PGF

A 100 μg/mL PGF methanol solution was analysed with a Dionex Ultimate 3000 high-performance liquid chromatography (HPLC) System (Thermo Fisher Scientific, Waltham, USA) coupled with a diode array ultraviolet/visible (UV–VIS) detector in which a Merck Chromolith® Performance C18 reversed-phase column (4.6 × 100 mm, 2 μm) column was used and eluted with a gradient mixture (from 20 to 70%) of an acetonitrile in 0.1% formic acid solution. Three components in the PGF fraction were identified with electrospray ionization mass spectrometry (ESI-MS) instrument from Shimadzu with an interface temperature of 300 °C and heating gas flow of 10 L/min. Data were collected in centroid mode from 100 to 1000 m/z.

### Total flavonoid content determination

The prepared fractions and rutin, as a standard (purchased from Hangzhou Huadong Medicine Group Wufeng Pharmaceutical Co., Ltd.), were dissolved in 70% ethanol and mixed successively with 1 mL of a 5% sodium nitrite solution, 1 mL of a 10% aluminium nitrate solution, and 10 mL of a 4% sodium hydroxide solution. Finally, the volume of each mixture was adjusted to 25 mL with 70% ethanol. The absorbance (*A*_510_) of the mixtures was measured at 510 nm over 15 min.

### Determination of antibacterial activity

The fractions and isolated components were separately dissolved in DMSO or ddH_2_O (water-soluble fraction) to a final concentration of 10 mg/mL, and the solutions were first subjected to susceptibility screening against bacterial strains with disc diffusion assays [17]. Whatman filter paper discs (diameter 6 mm) were impregnated with different fraction solutions as well as with both DMSO and ddH_2_O as solvent controls. These discs were placed on an MH broth agar plate containing 10^6^–10^7^ CFU/mL test strains. The plates were incubated at 37 °C for 24 h. The susceptibility was recorded by measuring inhibition zone diameters (IZDs) resulting from the growth inhibition around the discs.

### MIC and MBC identification

A 96-well microtiter plate and microbroth dilution method was used to determine the minimum inhibitory concentration (MIC), as previously described [18]. Each well containing 1 × 10^5^ to 1 × 10^6^ CFU/mL bacteria in MH broth medium (200 μL) was incubated at 37 °C for 24 h with 10 μL of test solutions, which were diluted serially at a 1:5 ratio (concentrations from 10 mg/mL to 1.25 μg/mL). Vancomycin and DMSO were used as positive and negative controls, respectively. The growth of bacteria was monitored by a SpectraMax 190 Microplate Reader (purchased from Molecular Devices) at 600 nm. For the minimum bactericidal concentration (MBC) determination, 10 μL aliquots from wells were plated on an MH agar plate and grown at 37 °C overnight. The MBC was recorded as the lowest concentration resulting in zero bacterial clones on the plate. Six repeats were performed for each well of the bacteria.

### Kinetic time-killing curve

A kinetic time-kill experiment was performed based on a modified method of Segovia et al. [19, 20]. Two standard *S. aureus* strains were separately grown in MH broth medium with a final count of approximately 1 × 10^5^ CFU/mL. The test solution was added into the broth culture to final concentrations of 1×, 2×, 4× and 8 × MIC. The bacteria cultured with an equivalent volume of DMSO or 8 μg/mL vancomycin were grown as negative and positive controls, respectively. The cultures were grown at 37 °C in a 180 rpm/min shaker. The cell concentration was determined by withdrawing 100 μL aliquots at 0, 3, 6, 10, and 20 h and plating onto MH agar plates on which the surviving bacteria could be counted overnight.

### Postantibiotic effect (PAE)

The postantibiotic effect represents a persistent suppression of bacterial growth after 1 h of exposure of bacterial cells to the PGF. First, 1 × 10^8^ CFU/mL freshly grown cells were incubated with 63, 125, and 250 μg/mL PGF in MH medium at 37 °C for 1 h. The cultures were diluted 1:1000 in pre-warmed MH medium and grown at 37 °C for 24 h. Viable bacterial counts were assessed at intervals of 0, 2, 4, 6, 8 and 24 h. The PAE was calculated as previously described [21].

### Cell cytotoxicity

NCTC 1469 cells (derived from mouse liver cells, obtained from the American Type Culture Collection) were seeded at a density of 2 × 10^4^ cells/well in Dulbecco’s modified Eagle medium (DMEM) (Sigma-Aldrich) containing 10% (v/v) foetal bovine serum (Sigma-Aldrich), 2 mM glutamine (Sigma-Aldrich), 5 U/mL penicillin (Sigma-Aldrich), and 50 μg/mL streptomycin (Sigma-Aldrich) and incubated at 37 °C in a humidified O_2_/CO_2_ (95:5) atmosphere overnight. On the second day, the cells were incubated in fresh cell medium containing different concentrations of the PGF and S3 under identical conditions for 16 h. After the corresponding treatments, the medium was removed, and cell viability was evaluated with the MTT method. The MTT assay kits were supplied by Sigma Chemical Co. (St. Louis, MO, USA). Mitochondrial dehydrogenases in live cells catalyse the reduction of MTT to a formazan salt, as described previously [22]. This reduced product presents a purple colour, whose absorbance can be measured with a plate reader at 510 nm.

### Statistics analysis

All data are presented as the mean ± SD. Statistical analyses were performed using one-way ANOVA, with a value of *p* < 0.05 indicating significant differences between treatments.

## Results

### PCP fraction preparation and total flavonoid content determination

After extraction, 250 g of PCP stem powder yielded 1.60 ± 0.03 g of petroleum ether (PEF), 8.43 ± 0.9 g of ethyl acetate (EAF), 5.80 ± 0.11 g of 1-butanol (BuOHF), and 18.18 ± 1.99 g of water (WF) fractions. The weight percentages of these four fractions were 0.64, 3.37, 2.32, and 7.27% (g/g stem powder), respectively. The total flavonoid contents of PEF, EAF, BuOHF, and WF were 5.23, 16.05, 7.58, and 5.73% (g/g), respectively. The PGF, which was eluted by 80% ethanol from the HPD 500 column, was the antibacterial fraction. The weight percentage of the PGF in the EAF was 73.39%, and the proportions of the three compounds S1, S2 and S3 were 6.01 ± 0.63%, 18.25 ± 2.02%, and 0.68 ± 0.10%, respectively, in the EAF.

### PGF component characterization

The components in the PGF fraction were analysed by an HPLC system coupled with a UV monitor (Fig. 1). The major components, S1 (Rt = 17.94 min), S2 (Rt = 20.22), and S3 (Rt = 22.13 min), were identified with HPLC combined with ESI-MS. The masses of S1, S2 and S3 were *m/z* 719, 871, and 873 (M-H)^−^, which were identical to those of known components in PCP: pinocembrin-7-O-[4″, 6″-hexahydroxydiphenoyl]-β-D-glucose (PHG), pinocembrin-7-O-[3″-O-galloyl-4″,6″-(s)- HHDP]-β-D-glucose (PGHG), and Thonningianin A [23].

**Fig. 1:** HPLC analysis of the PGF from PCP. First, 10 μL of the PGF (10 mg/mL) was analysed with a C18 reversed-phase column (Dionex). The process was monitored by a 254 nm UV detector. The Rt values of S1, S2 and S3 were 17.94, 20.22 and 22.13 min, respectively

### Antibacterial activity screening

The antibacterial activity of each fraction from PCP was initially screened by a disc diffusion assay with standard strains, *S. aureus* ATCC 29213, *S. aureus* ATCC 43300, *S. aureus* ATCC 25923, *S. epidermidis* CMCC 26069, *B. subtilis* CMC1.1470, *S. thermophilus* ATCC 19258, and *L. rhamnosus* ATCC 53103. The EAF, BuOHF, and PGF presented high efficiency against the tested bacteria, including three *S. aureus* strains, but the PEF and WF did not. The inhibition zone diameters (IZDs) are listed in Table 1.

**Table 1:** IZDs (mm) of different fractions of PCP extracts

Standard Strains	Fractions (10 mg/mL)				PGF (5 mg /mL)	Van (10 μg /mL)
	PF	EAF	BuOHF	WF		
*S. aureus* ATCC 29213	**–**	8.33 ± 0.58	6.83 ± 0.29	**–**	7.80 ± 0.30	23.85 ± 0.43
*S. aureus* ATCC 43300	**–**	10.75 ± 0.35	6.50 ± 0.71	**–**	8.38 ± 0.60	26.23 ± 0.31
*S. aureus* ATCC 25923	**–**	9.67 ± 0.82	6.67 ± 0.52	**–**	8.00 ± 0.26	27.35 ± 0.25
*S. epidermidis* CMCC26069	**–**	9.33 ± 0.58	6.67 ± 0.58	**–**	7.86 ± 0.69	Nd
*B. subtilis* CMCC 1.1470	**–**	10.83 ± 0.98	6.33 ± 0.52	**–**	8.80 ± 1.30	Nd
*S. thermophilus* ATCC 19258	**–**	10.50 ± 0.71	6.50 ± 0.71	**–**	7.33 ± 0.52	Nd
*L. rhamnosus* ATCC 53103	**–**	12.67 ± 0.58	6.33 ± 0.58	**–**	12.00 ± 0.83	Nd

Note: In the experiment, DMSO- and water-impregnated paper discs were used as negative controls. “-” indicates that no visible inhibition zone was observed. “Nd” means not detected

Anti-MRSA activity was determined with 7 clinical strains that were isolated from burn patients in the Surgery Department of Ningbo No. 2 Hospital from July to December 2017. The PGF presented antibacterial activity against all the tested MRSA strains, and the IZDs were between 8.1 and 11.2 mm. The multidrug-resistant properties and IZDs of each strain are listed in Table 2.

**Table 2:** IZDs (mm) of the PGF against different MRSA strains

Clinical Strains	Resistant (R)	Susceptible (S)	Intermediate (I)	IZDs
MRSA 170925062	CLI, CIP, CN, LEV, OX, PEN, SXT, TE, E, MXF	F, VAN, LZD, QD, TGC	RD	9.0 ± 0.35
MRSA 925059	OX, PEN	CLI, CIP, CN, TE, F, LEV, RD, SXT, VAN, E, MXF, LZD, QD, TGC	–	9.1 ± 0.43
MRSA 920057–1	CLI, CIP, CN, LEV, OX, PEN, SXT, TE, E, MXF	F, VAN, LZD, QD, TGC	RD	9.0 ± 0.74
MRSA 912036–2	CLI, CIP, CN, LEV, OX, PEN, SXT, TE, E, MXF	F, VAN, LZD, QD, TGC	RD	8.1 ± 0.43
MRSA 912037	CLI, CIP, CN, LEV, OX, PEN, SXT, TE, E, MXF	F, VAN, LZD, QD, TGC	RD	11.2 ± 0.76
MRSA 1223064–1	CLI, CIP, LEV, OX, PEN, SXT, TE, E, MXF	F, CN, VAN, LZD, QD, TGC	RD	10.4 ± 0.43
MRSA 1224057–1	CLI, CIP, LEV, OX, PEN, E, MXF	F, CN, VAN, LZD, QD, TGC, TE, RD, SXT	–	10.1 ± 0.75

Note: “-” indicates that no visible inhibition zone was observed

*Abbreviations*: *CIP* Ciprofloxacin, *CLI* Clindamycin, *CN* Cephalexin, *E* Erythromycin, *F* Nitrofurantoin, *LEV* Levofloxacin, *LZD* Linezolid, *MXF* Moxifloxacin, *OX* Oxacillin, *PEN* Penicillin, *QD* Quinupristin/dalfopristin, *RD* Rifampicin, *SXT* Sulfamethoxazole/trimethoprim, 19:1, *TE* Tetracycline, *TGC* Tigecycline, *VAN* Vancomycin

### MIC and MBC determination

The antibacterial activity of the PGF, S1, S2, and S3 was evaluated with MICs, MBCs, and MBC/MIC ratios in this study. Interestingly, the PGF and three isolated components could inhibit the growth of the two tested strains with an MIC of 62.5 μg/mL. However, the PGF and S3 presented the best killing activity against *S. aureus*, and the MBC/MIC ratios were between 2 and 4. The MBC and MIC of vancomycin, the positive control, against each strain were 2 μg/mL, and the MBC/MIC ratio was 1. The results are listed in Table 3.

**Table 3:** MICs and MBCs of the PGF, S1, S2, and S3

MICs, MBCs and MIC/MBC ratios of the active fraction, components and vancomycin (μg/mL)	Test strains	
	*S. aureus* ATCC 25923	*S. aureus* ATCC 43300
PGF		
MIC	62.5	62.5
MBC	125	250
MBC/MIC	2	4
S1		
MIC	62.5	62.5
MBC	–	–
MBC/MIC	–	–
S2		
MIC	62.5	62.5
MBC	–	500
MBC/MIC	–	8
S3		
MIC	62.5	62.5
MBC	250	250
MBC/MIC	4	4
Vancomycin		
MIC	2	2
MBC	2	2
MBC/MIC	1	1

Note: “-” indicates the value could not be identified

### Kinetic time-kill curve

The bactericidal/bacteriostatic activities of the PGF and S3 were determined with a time-kill experiment. First, 1 × MIC of the PGF produced a weak killing efficiency against *S. aureus* ATCC25923, as it was shown that approximately 2 logs (CFU/mL) of the bacteria were killed in 20 h. In comparison, an evident killing efficiency of 2 × MIC and 4 × MIC was observed in 6 h. For *S. aureus* ATCC 43300, as high as 4 × MIC of the PGF could kill most of the bacteria, more than 4 logs (CFU/mL), in 6 h (Fig. 2). The bactericidal activity of 8 × MIC and 4 × MIC S3 could be detected in 24 h (against strain ATCC 25923 and ATCC 43300, respectively). Strain ATCC 43300 was more susceptible to S3 than ATCC 25923 (Fig. 3). Two logs (CFU/mL) of ATCC 43300 bacteria were killed in 3 h with 4× and 8 × MIC S3. In comparison, 1 log (CFU/mL) of ATCC 25923 bacteria was killed in 3 h with 4× and 8 × MIC S3.

**Fig. 2:** Time-dependent killing activities of the PGF on strains ATCC 25923 and ATCC 43300. All the CFU values are the average of 6 repeats

**Fig. 3:** Time-dependent killing activities of S3 on the strains ATCC 25923 and ATCC 43300. All the CFU values are the average of 6 repeats

### Postantibiotic effect (PAE) of the PGF

Postantibiotic effects are one of the antibiotic properties that are affected by bacterial species. The PAEs of 1 × MIC, 2 × MIC, and 4 × MIC (63, 125 and 250 μg/mL, respectively) the PGF on strain ATCC 25923 were 1.47, 1.49, and 1.94 h, respectively. However, the PAEs of the PGF on strain ATCC 43300 were dose-dependent (*p* < 0.05), which were 0.28 (1 × MIC), 1.13 (2 × MIC), and 4.68 (4 × MIC) h. This result is listed in Table 4 in detail.

**Table 4:** Postantibiotic effects of the PGF

Con. of the PGF	Mean of PAE ± st (h)	
	*S. aureus* ATCC 25923	*S. aureus* ATCC 43300
63 μg/mL	1.47 ± 0.30	0.28 ± 0.17
125 μg/mL	1.49 ± 0.36	1.13 ± 0.16
250 μg/mL	1.94 ± 0.45	4.68 ± 0.87

### Cytotoxicity of the PGF and S3

To study the cytotoxicity of the PGF, we evaluated NCTC 1469 cell (from the American Type Culture Collection, Manassas, VA) viability with an MTT assay after drug treatment. As shown in Fig. 4, inclusion of the PGF in the medium caused dose-dependent decreases in the relative MTT levels. Although 400 μg/mL caused a slight decrease in cell viability, this concentration was much higher than 4 × MIC the PGF. NCTC cells were more sensitive to S3 (< 80 μg/mL) than to the PGF. This result suggested that the PGF but not S3 was more toxic to *S. aureus* than to eukaryotic cells.

**Fig. 4:** Influence of the PGF and S3 on cell viability. The PGF decreased cell viability in a dose-dependent manner, as shown by the MTT assay. NCTC 1469 cells were incubated with increasing concentrations of the PGF or S3 for 18 h. * * *P* < 0.01 vs. UT (0 μg/mL). UT indicates an untreated control

## Discussion

In this study, the crude extract of PCP stems was separated into 4 fractions, the PEF, EAF, BuOHF, and WF, by a liquid-liquid partitioning extraction method. The bacteriostatic activity of each fraction was identified with the IZD method. The EAF presented the most significant antibacterial activity (Table. 1). Furthermore, we separated the EAF with an HDP 500 column using 30% ethanol to flow through, 80% ethanol to elute (PGF), and 95% ethanol to wash the column. The PGF presents high antibacterial activities against MRSA strains (Table. 2).

The components in the PGF were characterized by HPLC (Fig. 1). The molecular masses of three components were identified with LC-MS. Based on the molecular masses, we concluded that the three main components, S1, S2, and S3, were pinocembrin-7-O-[4″, 6″-hexahydroxydiphenoyl]-β-D-glucose, pinocembrin-7-O-[3″-O-galloyl-4″,6″-(s)-hexahydroxydiphenoyl]-β-D-glucose, and pinocembrin dihydrochalcone-7-O-[3″O-galloyl-4″,6″-hexahydroxydiphenoyl]-β-D-glucoside (Thonningianin A), respectively. These compounds are ellagitannins composed of pinocembrin (or dihydrochalcone), hexahydroxydiphenic acid, and gallic acid (in S2 and S3) linked to a glucose molecule. Pinocembrin commonly exists in a variety of plants [24, 25] and bee products, such as honey [26] and propolis [27]. Hexahydroxydiphenic acid, whose galloyl groups are linked through C-C bonds, is found in different fruits, e.g., strawberries, raspberries, and blackberries [28]. Gallic acids are present in various plants [29–31] However, S1, S2, and S3 are not commonly distributed molecules in plants. Thonningianin A (S3) was isolated from *Thonningia sanguinea* decades ago [32] The antibacterial activity of *Thonningia sanguinea* extract was explored [17]. S1 was isolated from *Stylogne cauliflora* and identified by Hegde and Chan in 2003 [33], which presents anti-viral activity [34]. S2, structurally similar to S3, is specific in PCP [34].

Next, the bacteriostatic and bactericidal activities of the PGF as well as of S1, S2, and S3 against *S. aureus* were identified quantitatively. The MICs of the PGF and the three compounds on standard strains were 63 μg/mL (Table 3), which is identical to that of berberine, a clinically used medicine [35]. No bactericidal activity of S1 was observed (Table 3). S2 could kill only strain 43,300, with an MBC/MIC ratio of 8. The MBC/MIC ratio of S3 on both *S. aureus* strains was 4. Generally, an MBC/MIC ratio less than 2 is considered bactericidal for an antibiotic, and an MBC/MIC> 8 is indicative of bacteriostatic behaviours [36, 37]. Therefore, we proposed that S3 is the key efficacious molecule in the PGF. The bactericidal/bacteriostatic behaviour of the PGF and S3 was confirmed by time-kill assays (Figs. 3 and 4). Notably, in comparison to the efficiencies of S1 and S2, that of the PGF presented faster and stronger bactericidal activity than S3.

Both antibiotics and disinfectants could possibly affect cell processes, e.g., the substrate transport systems and cell wall or DNA synthesis processes, after a brief exposure of bacteria to a low dose of drugs. This phenomenon is called the postantibiotic effect (PAE). The PAE can be influenced not only by the duration of exposure, bacterial species, and culture medium but also by the class of antibiotics. In this study, the PAE of the PGF against ATCC 43300 but not against ATCC 25923 was dose dependent. This result could be due to different potential mechanisms that still need to be studied deeply. Both strains could form biofilms, and only ATCC 43300 was a MRSA strain [38]. It seems that ATCC 43300 was more susceptible than ATCC 25923 to S2 and S3. We proposed that S3 or the PGF from PCP may be a good candidate for a bactericide.

For clinical application, no cytotoxic effect is expected. However, the components composing herbal extracts are generally a complex of phenolics, flavonoids, or alkaloids. All these components may also influence the viability of normal eukaryotic cells. It is important to demonstrate the cell safety of the PGF. No significant cytotoxicity of the PGF (Con. < 600 μg/mL) was observed in an in vitro NCTC cell assay. In contrast, S3 was more toxic to eukaryotic cells than to bacteria (Fig. 4).

## Conclusions

The PGF, an extract fraction of *Penthorum chinense* Pursh, presents anti-*S. aureus* MRSA activity, which is one of the contaminants that causes skin infections. This activity may be a coordinated action of three components, pinocembrin-7-O-[4″,6″-hexahydroxydiphenoyl]-β-D-glucose, pinocembrin-7-O-[3″-O-galloyl-4″,6″-(s)-HHDP]-β-D -glucose (PGHG) and Thonningianin A.

## Data Availability

All data described in this manuscript are available from the corresponding author on reasonable request.

## Abbreviations

CFU: Colony-forming units
DMSO: Dimethyl sulfoxide
ESI-MS: Electrospray ionization mass spectrometry
HHDP: Hexahydroxydiphenoyl
HPLC: High-performance liquid chromatography
IZDs: Inhibition zone diameters
MBC: Minimum bactericidal concentration
MH: Mueller-Hinton
MIC: Minimum inhibitory concentration
MRSA: Methicillin-resistant *Staphylococcus aureus*
MTT: 3-(4,5-dimethylthiazol-2-yl)-2,5-diphenyltetrazolium bromide
PAEs: Postantibiotic effects
PCP: *Penthorum chinense* Pursh
PGF: Pinocembrin-7-O residue-rich fraction in PCP
UV–VIS: Ultraviolet/visible
